The article "White-Light Endoscopic Colorectal Lesion Detection Based on Improved YOLOv5" was published in 2022. Journal: Comput Math Methods Med.

# White-Light Endoscopic Colorectal Lesion Detection Based on Improved YOLOv5

**DOI:** 10.1155/2022/9508004

**Published:** 2022-01-22

**Authors:** Junbo Gao, Qilin Xiong, Chang Yu, Guoqiang Qu

**Affiliations:** ^1^Information Engineering College, Shanghai Maritime University, Shanghai 201306, China; ^2^Department of Gastroenterology, Eastern Hospital, Shanghai Sixth People Hospital, Shanghai 201306, China

## Abstract

As an effective tool for colorectal lesion detection, it is still difficult to avoid the phenomenon of missed and false detection when using white-light endoscopy. In order to improve the lesion detection rate of colorectal cancer patients, this paper proposes a real-time lesion diagnosis model (YOLOv5x-CG) based on YOLOv5 improvement. In this diagnostic model, colorectal lesions were subdivided into three categories: micropolyps, adenomas, and cancer. In the course of convolutional network training, Mosaic data enhancement strategy was used to improve the detection rate of small target polyps. At the same time, coordinate attention (CA) mechanism was introduced to take into account channel and location information in the network, so as to realize the effective extraction of three kinds of pathological features. The Ghost module was also used to generate more feature maps through linear processing, which reduces the stress of learning model parameters and speeds up detection. The experimental results show that the lesion diagnosis model proposed in this paper has a more rapid and accurate lesion detection ability, and the AP value of polyps, adenomas, and cancer is 0.923, 0.955, and 0.87, and mAP@50 is 0.916.

## 1. Introduction

Colorectal cancer (CRC) has become the most common gastrointestinal malignancy in the world after male prostate cancer, female breast cancer, and lung cancer [1]. However, patients with early colorectal cancer do not show obvious clinical symptoms. When using white-light endoscopy for detection, it is easy to miss the detection of lesions due to the influence of doctors' operation level, subjectivity, fatigue, and other factors [2], thus leading to the missing of the best treatment opportunity for patients in the middle and late stages. Combining white-light endoscopy with computer-aided diagnosis (CAD) can reduce the rate of missed diagnosis caused by physician judgment alone, thus improving the survival rate of colorectal cancer patients [3, 4]. At present, there are two methods for computer-aided detection of colorectal lesions: one is based on traditional machine learning, and the other is based on deep learning. The most important step is to extract the features of colorectal lesions.

Traditional methods use simulation to distinguish low-level features to determine the likelihood of colorectal lesions, for example, shape feature-based [5], texture feature-based [6], and valley depth-based [7]. However, due to intragroup variation, colorectal lesions have different sizes, shapes, edge textures, and distributions. When using a white-light endoscope, the surface of the colonic mucosa was reflective. The feature extraction is also prone to interference from intestinal contents (foam, manure water, dung residue, etc.), so the manual method based on traditional machine learning is unreliable and time-consuming, which is not enough to extract the complex pathological features in the intestinal tract.

The article "White-Light Endoscopic Colorectal Lesion Detection Based on Improved YOLOv5" was published in 2022. Journal: Comput Math Methods Med.

Deep learning uses the hierarchical feature learning ability of convolutional neural network to detect colorectal lesions, and its detection methods can be divided into two-stage detection and one-stage detection. Due to the high accuracy obtained by the two-stage target detection algorithm at the cost of the detection speed and the large amount of computation, it is not suitable for real-time detection and is not widely applied in equipment with insufficient computing power. Therefore, this paper pays more attention to the benefits of the one-stage detection model in the diagnosis of colorectal lesions. A relevant study [8] proved the feasibility of YOLO algorithm in assisting the diagnosis of lesions. The localization accuracy of the algorithm for lesions reached 79.3%, the sensitivity reached 68.3%, and the detection efficiency was 0.06 seconds/frame. In the study conducted by [9], a regression-based ResYOLO convolutional neural network was proposed, and the detection accuracy, recall rate, and detection speed of polyps were 88.6%, 71.6%, and 6.5 frames/sec, respectively. In the study [10], YOLOv3 algorithm was used to detect gastric polyps, and small polyps were detected from the background as the breakthrough direction. The accuracy and recall rate of this method reached 91.6% and 86.2%, respectively.

To sum up the above, the effective detection of colorectal lesions can reduce the incidence of colorectal cancer. It is difficult for the traditional machine learning method to accurately detect the complicated intestinal lesions. Deep learning-based YOLO algorithm has potential for colorectal lesion detection, but most of the articles are aimed at diagnosing only a single polyp lesion. Colorectal cancer is stage-specific, going through a series of changes from polyps and adenomas to cancer. The doctor can only recommend a targeted treatment plan if it takes into account the patient's specific type of lesion. Therefore, this study positioned the diagnosis of colorectal lesions as three-category lesion detection and made full use of the advantages of the YOLO algorithm. Based on YOLOv5 [11], Mosaic data enhancement strategy was adopted to improve the detection ability of micropolyps. The CA mechanism [12] was introduced into the feature extraction network structure to enhance the model's effective attention to the three lesion types. At the same time, Ghost module [13] was introduced to reduce the number of parameters in ordinary convolution calculation to accelerate the processing speed of colorectal lesion detection.

The article "White-Light Endoscopic Colorectal Lesion Detection Based on Improved YOLOv5" was published in 2022. Journal: Comput Math Methods Med.

## 2. Materials and Methods

This paper proposes a modified YOLOv5-based colorectal lesion detection model YOLOv5x-CG, and the research process is shown in Figure 1. Data preprocessing was first performed, including both data enhancement and data annotation. Then, preset the initial anchor boxes. The dashed box shows the improved YOLOv5 lesion diagnosis model, and the details of which will be described later. Finally, the model was evaluated with the validation data set and lesions were predicted on the test set.

### 2.1. The Data Processing

In response to the small amount of available data and the uneven distribution of the various lesion categories, this paper expands the lesion sample data. The basic experimental data in this paper were provided by Digestive Endoscopy Center, Lingang Hospital, Shanghai Sixth People's Hospital, China, and were based on the images of colorectal lesions detected by white-light endoscopy (as shown in Figure 2(a)). The time dimension of patient data was from June 2015 to September 2019. After screening the data without lesion targets, a total of 1709 original lesion data were obtained for the experiment. The image size used in the experiment was 420 × 389 × 3 (RGB). During data enhancement, we performed basic operations such as rotating and flipping the original image; in addition, while keeping the hue basically unchanged, we combined the HSV color space [14] to perform the saturation and lightness of the image fine-tuned. The enhancement effect is shown in Figure 2(b).

In particular, HSV color enhancement is intended to simulate the different light intensities that may occur during white-light endoscopic operations, where different types of colorectal lesions have different color characteristics, thus improving the generalisation of the model during training. Through a series of data enhancement operations, the data set was expanded to 4949 pieces, including three lesion categories: polyps, adenomas, and colorectal cancer.

In this paper, LableImg image data annotation software was used to annotate the outer rectangular box of the lesion target. We tried to ensure that the surrounding target area contains as little intestinal background information as possible. During the process, the annotation files are stored in the YOLO format. The image and the corresponding annotation files are divided into a training set, validation set, and test set through Python code, and their ratios in the enhanced data set are, respectively, 8 : 1 : 1. The data distribution of each lesion category is shown in Table 1.

The article "White-Light Endoscopic Colorectal Lesion Detection Based on Improved YOLOv5" was published in 2022. Journal: Comput Math Methods Med.

### 2.2. Preset Anchor Box

In order to make the model better locate the position of colorectal lesions in the regression stage of boundary boxes, this paper presets the anchor box based on *k*-means clustering algorithm [15] combining the information of the real annotation boxes of lesions.  Figure 3 shows the distribution of the center point and lesion size of the lesion target in the data set relative to the original image. Both (a) and (b) in Figure 3 show the distribution after normalization.

It can be found that the distribution of lesion target centers is relatively uniform, and a few lesion centers are concentrated near the image center. A considerable number of lesions are concentrated in the small target category. Therefore, this paper combines *k*-means algorithm to complete the following steps to preset the anchor boxes.

**Step 1 .**

Extract the coordinate information of all the annotation boxes.

**Step 2 .**

Obtain the height and width data of the annotation box through the corresponding coordinate information.

**Step 3 .**

Randomly select 9 annotation boxes as the starting values of anchors.

**Step 4 .**

Each annotation box performs IoU operation with these 9 randomly selected anchors, using *d* = 1 − IoU as a distance measure. The greater the *d*, the greater the error between the two.

**Step 5 .**

Categorization: for a given annotation box, place it in the category of the anchor with which it has the smallest *d* value.

**Step 6 .**

After all the annotation boxes have been grouped, the height and width of all the annotation boxes in the 9 anchors' category are averaged to obtain the updated 9 anchors.

**Step 7 .**

Repeat Step 4-6, and stop the clustering operation when the position of the annotation boxes in the 9 anchors category no longer changes.

**Step 8 .**

Output the 9 anchor boxes obtained by clustering.

IoU is the intersection and union ratio of the annotation box and the anchor box. The image size of the colorectal lesion used in this paper is 420 × 389 × 3. In order to meet the image size requirements of the model, the letterbox function adjusted the input image to 448 × 448 × 3 by resize and then padding. The initial anchor boxes obtained by the final clustering are shown in Table 2.

The article "White-Light Endoscopic Colorectal Lesion Detection Based on Improved YOLOv5" was published in 2022. Journal: Comput Math Methods Med.

## 3. Model Construction

### 3.1. Model Introduction

In order to realize the flexible deployment of the model and improve the feasibility of project implementation, this paper combines the target detection YOLOv5 algorithm for the construction of colorectal lesion diagnosis model, which mainly consists of the following three parts, and the specific network details are shown in Figure 4:

1. Backbone: it consists of Focus, Conv, SPP, CA, and other modules to realize the extraction of features from the input image. The Focus module slices the image; after the Focus module, the original 448 × 448 × 3 image first becomes a 224 × 224 × 12 feature map. Because the Focus module has 80 convolution kernels, the convolution operation is performed through 80 convolution kernels and finally obtained a feature map of 224 × 224 × 80. The Focus module can reduce the cost of convolution operation and reduce the loss of information; the Conv module consists of Conv2d with the BN (Batch Normalization) [16] layer and the SILU activation function; the SPP [17] module performs maximum pooling at three different scales, fusing features from feature maps of different sizes to increase the perceptual field while reducing the loss of lesion features, where the CA module is described in detail in Section 3.3
2. Neck: improve detection performance, which combines the ideas of FPN [18] and PANET [19]; the FPN module transfers rich semantic features from the top layer to the bottom layer, and the PANET module effectively transfers the localization features from the bottom layer to the top layer by extending the bottom-up path, thus improving the detection capability for lesion targets of different sizes
3. Detect: localization and classification of detection targets. Three vectors will be output in the detection network, and each output vector has the predicted values of three anchor boxes, which are used to detect targets of different sizes

### 3.2. Mosaic Data Enhancement Strategies

Early polyps with small target features, especially small flat polyps, are extremely easy to miss. In response to this phenomenon, this paper combined the Mosaic data enhancement strategy proposed in YOLOv4 [20] to randomly select four white-light endoscopy images participating in the training during the training model and recombine them into a complete large image, as shown in Figure 5.

The Mosaic data enhancement strategy approach allows otherwise smaller polyp elements to be detected in a smaller field of sensation, thereby increasing the detection rate of small target polyps.

### 3.3. Improvement of Feature Extraction Network

In order to highlight the different contributions of each region in the feature map to the detection results, different attention is applied to each feature point so that more colorectal lesion features are effectively extracted. In this paper, coordinate attention (CA) [12] is introduced to capture the relationship between location information and each channel in the feature extraction network structure. The embedding process of coordinate information decomposes the global average pooling in SENET [21] into two one-dimensional feature encodings for the aggregation of spatial features along *x* and *y* directions.

(1) $$\begin{array}{c} Z_{c}=\frac{1}{H\times W}\overset{H}{\underset{i=1}{\sum }}\overset{W}{\underset{j=1}{\sum }}x_{c}\left(i,j\right). \end{array}$$

The meaning of the global average pooling formula (1) is to output a value after global averaging of a feature map; i.e., an *H* × *W* × *D* tensor becomes a 1 × 1 × *D* tensor after global average pooling.

(2) $$\begin{array}{c} Z_{c}^{h}\left(h\right)=\frac{1}{W}\underset{0\leq i<W}{\sum }x_{c}\left(h,i\right), \end{array}$$

(3) $$\begin{array}{c} Z_{c}^{w}\left(w\right)=\frac{1}{H}\underset{0\leq j<H}{\sum }x_{c}\left(j,w\right). \end{array}$$

Equations (2) and (3) indicate that for input *X*, each channel is encoded using pooling kernels (*H*, 1) along the horizontal direction and pooling kernels (1, *W*) along the vertical direction, respectively

(4) $$\begin{array}{c} f=\delta \left(F_{1}\left(\left[Z^{h},Z^{W}\right]\right)\right). \end{array}$$

*F* in (4) denotes the Concat operation, and *f* denotes the intermediate feature mapping after BN using the nonlinear activation function *σ* to obtain the horizontal and vertical directions after encoding.

(5) $$\begin{array}{c} g^{h}=\sigma \left(F_{h}\left(f^{h}\right)\right), \end{array}$$

(6) $$\begin{array}{c} g^{w}=\sigma \left(F_{w}\left(f^{w}\right)\right). \end{array}$$

Equations (5) and (6) denote the decomposition of *f* into tensor *f*^*h*^ and tensor *f*^*w*^ along the spatial dimension and then the convolutional transformation of *F*_*h*_ and *F*_*w*_ so that *f*^*h*^ and *f*^*w*^ have the same number of channels, where *σ* denotes the sigmoid activation function, and the final attention weights are generated from (7). The network structure of this module is shown in Figure 6.

(7) $$\begin{array}{c} y_{c}\left(i,j\right)=x_{c}\left(i,j\right)\times g_{c}^{h}\left(i\right)\times g_{c}^{w}\left(j\right). \end{array}$$

In this paper, we make full use of the superiority of this module on mobile networks with insufficient computational overhead capacity by connecting a CA module after the ordinary convolutional layer and SPP module of the feature extraction network structure, and the number of convolutional kernels used in the added CA module is 160, 320, 640, and 1280, respectively. This allows a better remote dependence of the extracted features along the spatial direction without losing the location information, and the resulting attentional feature map adds attention to the lesion region based on the original input feature map, as shown in Figure 7. It can be found that the original network structure is extracted for global features, and the background gut information is instead more fine-grained, and the lesion location is given more attention after the CA module processing.

The article "White-Light Endoscopic Colorectal Lesion Detection Based on Improved YOLOv5" was published in 2022. Journal: Comput Math Methods Med.

### 3.4. Improvement of Feature Fusion Network

After adding the CA module, the network layer of the model changes from the original 607 layers to 815 layers. Although the number of parameters to be learned in the training process is reduced by about 27.8%, the overall network architecture still bears heavy computational pressure. Therefore, in this paper, the Ghost module proposed in [13] is used in the feature fusion phase to linearly expand some of the features extracted from the feature extraction network. As shown in Figure 8, the Ghost feature generation module (GFGM) first generates part of the feature graph (a) by the convolution operation and then makes a series of linear transformations from the feature graph(∅_1_, ∅_2_, ⋯, ∅_*j*_), gets its mapped feature graph (b), and finally splices (a) and (b) together for a specific dimension to obtain (c). The linear transformation ∅ operation used in this article is similar to the 5 × 5 convolution. With the use of this module, the number of parameters to be learned was reduced by 71.7% and the speed of detection was increased by 53.8% compared to the original network.

## 4. Model Training and Evaluation

### 4.1. Model Training

In our study, the learning rate was set to 0.01 to accelerate the model convergence. Secondly, Adam was selected for hyperparameter optimization, and the learning rate momentum was set to 0.95 in consideration of the small number of samples in the data set of colorectal lesions. Meanwhile, we use a pretrained model for training assistance, which can make the model have better initial performance. After 300-epoch training, the performance indicators tend to stabilize, and the training ends. The environment configuration used in the experiment is shown in Table 3.

### 4.2. Evaluation Indicators

In this study, the performance of the diagnostic model for colorectal lesions was evaluated by validating data sets and quantified by the following indicators:

(8) $$\begin{array}{c} P=\frac{\text{TP}}{\text{TP}+\text{FP}}, \end{array}$$

(9) $$\begin{array}{c} R=\frac{\text{TP}}{\text{TP}+\text{FN}}, \end{array}$$

(10) $$\begin{array}{c} \text{AP}=\int_{0}^{1}P\left(R\right)dR, \end{array}$$

(11) $$\begin{array}{c} \text{mAP}=\frac{1}{C}\overset{C}{\underset{i=1}{\sum }}\text{A}\text{P}\left(i\right), \end{array}$$

where *P* is accuracy rate and *R* is recall rate: true positive (TP) is the number of colorectal lesions correctly identified; false positive (FP) represents the number of misidentified colorectal lesions; false negative (FN) represents the number of missed colorectal lesions. AP is the average accuracy; *P*(*R*) is the accuracy *P* corresponding to different recall rates *R* and corresponds to the area under the *P*-*R* curve. In (11), *C* is 3, representing the three-lesion categories of polyps, adenomas, and cancer. mAP is the average number of APs in each category, where mAP@0.5 is the average AP of the three lesions when IoU is 0.5. mAP@0.5 : 0.95 is the average mAP on different IoU whose threshold value is between 0.5 and 0.95 and step size is 0.05. In addition, we also evaluate the model training parameters and network reasoning time.

The article "White-Light Endoscopic Colorectal Lesion Detection Based on Improved YOLOv5" was published in 2022. Journal: Comput Math Methods Med.

## 5. Results and Discussion

In order to verify the superiority of the diagnosis model of colorectal lesions under the combined action of CA module and Ghost module, we conducted 4 groups of comparison experiments. Experiment 1 is the original YOLOv5x network structure. In experiment 2, CA module was introduced. In experiment 3, Ghost module was introduced. Experiment 4 used the model proposed in this study, which introduces both the CA module and the Ghost module. The network structure name and structure distribution of each experiment are shown in Table 4. The same experimental operation was performed on these four model structures. Figures 9 and 10 and Table 5 recorded the changes of some indicators in different models and AP values of each lesion category in the experimental process.

Figure 9 represents the changes in the performance metrics of colorectal lesion detection for the four different network structures during training with an epoch set to 300. The metric changes tend to level off after an average of 80 epochs. The red curve represents YOLOv5x-CG network structure. Compared with the other three structures. It is almost at the highest level in terms of accuracy, recall, and mAP.

The final results of the model evaluation are shown in Table 5, where it can be seen that the original YOLOv5 model did not perform well in terms of accuracy, recall, and mAP and that although there was some improvement using either the CA module or the Ghost module alone, the overall performance was not as good as that of the YOLOv5x-CG network combining the two. The YOLOv5x-CG network structure of precision, recall, and mAP@50 improved by 7.4%, 1.5%, and 7.1%, respectively, compared to the original YOLOv5x.

The article "White-Light Endoscopic Colorectal Lesion Detection Based on Improved YOLOv5" was published in 2022. Journal: Comput Math Methods Med.

The AP values for the detection of polyps, adenomas, and cancer for each of the above four network structures are illustrated in Figure 10. It can be seen that YOLOv5x-CG performed well in terms of AP for adenomas and polyps, reaching 0.923 and 0.955, respectively, and the effective detection of adenomas and polyps is crucial for the prevention of colorectal cancer.

The analysis of the number of network layers, the number of parameters in the network, and the model inference speed for different structures is shown in Table 6. The results show that the YOLOv5x-CG proposed in this paper not only performs well in evaluation metrics such as mAP but also has fewer network parameters and faster model inference speed.

Finally, we used YOLOv5X-CG model weights to predict lesions in the test set, and the prediction results are shown in Figure 11. The location of each lesion basically fits the lesion itself, and the detection ability of small target polyps is almost equal to that of relatively large adenomas and cancers, and the missed detection, false detection, and low confidence score of original YOLOv5x prediction results are improved to some extent, as shown in Figure 12.

The upper panel of Figure 12 shows the partial detection of the original YOLOv5 and the lower panel shows the partial detection of YOLOv5x-CG, where (a) indicates that YOLOv5x-CG detects polyps missed by YOLOv5, (b) indicates that YOLOv5x-CG improves the confidence level of adenomas in YOLOv5, and (c) indicates that YOLOv5x-CG corrects polyps that were YOLOv5 misdetected cancer.

## 6. Conclusions

The strong strategy improves the detection of micropolyps, while the combination of CA attention module and cheap feature generation Ghost module effectively improves the detection rate and speed of detection of colorectal lesions. Since ordinary white-light endoscopy is used by many urban hospitals in China, the model proposed in this study can be better combined with white-light endoscopic imaging technology to give a more intelligent and efficient capability for the detection of colorectal lesions at different stages, thus reducing the burden of manual visits by physicians and effectively improving the lesion detection rate. The current work in this paper is more on improving the accuracy of the model. Due to the large memory occupied by the model and its dependence on the device, the model still needs to be compressed and accelerated during the actual deployment to better fit in the low-powered devices, which will be carried out in the next experiments.

The article "White-Light Endoscopic Colorectal Lesion Detection Based on Improved YOLOv5" was published in 2022. Journal: Comput Math Methods Med.

## Figures and Tables

**Figure 1:** Flow chart of the YOLOv5x-CG model for colorectal lesion detection.

**Figure 2:** (a) Shows the original white-light endoscopic image of the colorectal lesion. (b) Shows the image of the lesion after rotation, flipping, and HSV color enhancement.

**Figure 3:** (a) Distribution of central points of colorectal lesions. (b) Size distribution of colorectal lesions.

**Figure 4:** YOLOv5x-CG: network structure for colorectal lesion diagnosis.

**Figure 5:** Mosaic combination during model training.

**Figure 6:** CA module structure details.

**Figure 7:** Comparison of the different feature maps of the original network and the processed output of the CA module. (a) Shows the output feature map after processing of the original network structure. (b) Shows the map corresponding to the adenoma lesion in the input network. (c) Shows the output feature map after processing by the CA module.

**Figure 8:** Ghost feature generation (GFGM): (a) convolution operation to generate partial feature maps; (b) feature map generated by linear transformation; (c) feature map after splicing combination.

**Figure 9:** Variation of each metric for different network structures at 300 epochs.

**Figure 10:** AP values for each lesion category for different models.

**Figure 11:** YOLOv5x-CG model prediction result presentation.

**Figure 12:** Comparison of test results: (a) missed polyp; (b) increased confidence in adenomas; (c) misdiagnosed cancer.

**Table 1:** Data distribution of each lesion type.

Category	Polyps	Adenomas	Colorectal cancer	Total
Original	381	1048	280	1709
Expanded	1650	1655	1644	4949

**Table 2:** The initial anchor boxes.

Initial anchor box size		
72 × 69	91 × 96	116 × 122
172 × 150	159 × 214	240 × 208
251 × 311	331 × 303	391 × 361

**Table 3:** Experimental environment configuration.

Environment	Details
Processor	AMD Ryzen 7 4800H with Radeon Graphics
Operating system	Windows 10
Video cards	NVIDIA GeForce RTX 2060 6 GB
PyTorch version	Torch 1.8.1 + cu102

**Table 4:** Improved modules of different network structures.

Network structure	CA module	Ghost module
YOLOv5x	—	—
YOLOv5x-Ghost	—	Neck
YOLOv5x-CA	Backbone	—
YOLOv5x-CG	Backbone	Neck

**Table 5:** Presentation of the final results for each indicator for different network structures.

Network structure	Precision	Recall	mAP@50
YOLOv5x	0.799	0.825	0.845
YOLOv5x-CA	0.83	0.814	0.9
YOLOv5x-Ghost	0.816	0.869	0.874
YOLOv5x-CG	0.873	0.840	0.916

**Table 6:** Other performance comparisons for different networks.

Network structure	Network layer	Network parameters	Test reasoning speed
YOLOv5x	607	87257832	30.5 ms
YOLOv5x-Ghost	395	51703568	16.7 ms
YOLOv5x-CA	815	63040072	18.5 ms
YOLOv5x-CG	623	24693808	14.1 ms

The article "White-Light Endoscopic Colorectal Lesion Detection Based on Improved YOLOv5" was published in 2022. Journal: Comput Math Methods Med.

## Data Availability

The data used to support the findings of this study are available from the corresponding author upon request.
